# Machine-Vision-Based Intelligent Manufacturing by Fine-Grained Point Cloud Identification

This article has been retracted.

**DOI:** 10.1155/2022/5627959

**Published:** 2022-09-16

**Authors:** Yinhai Li, Fei Wang, Yang Jiang

**Affiliations:** ^1^College of Mechanical and Electrical Engineering, Jinhua Polytechnic, Jinhua 321007, Zhejiang, China; ^2^College of Creative Arts, Jinhua Polytechnic, Jinhua 321007, Zhejiang, China; ^3^Jinhua KEDI Instrumental Equipment Co. LTD, Jinhua 321007, Zhejiang, China

## Abstract

Traditional manufacturing system inspections are primarily conducted through microtools. Nowadays, the size of consciously manufactured parts that is getting smaller and smaller, wherein unwritten methods are subject to subjectivity, often resulting in reckless deviations. It is necessary to develop a highly efficient and correct discovery technique. Given the leaned flexibility of traditional manufacturability analysis methods based on cognitive notoriety and empire foundation, the reality that existing manufacturability analysis methods based on full scientific support cannot give a specific purpose for capability manufacturability. A deep cognition support framework grants the manufacturability analysis example. Manufacturing separative methods are presented as imitate. First, a large enumeration of 3D CAD plan with specific manufacturability are made by digital modeling technology, wherein the tier genealogy is realized to cause the data adjustments required for thorough academics. Then, concavity-oriented designs are established on the PointNet entangle form manufacturability. Dense learned grids were analyzed, and network parameter tuning and management were done; then comparisons with voxel-representation-enabled three-dimensional convolutional neural networks (3D-CNN) and existing methods revealed detailed literature for fabricating networks with better robustness and lower algorithm cycle complexity; finally, the actual completion of the network is verified through the example section, and the manufacturability of the cave shape is analyzed to identify the unmanufacturable overall form and explain its considerations. The experimental results have shown that the rule can determine the specific reasons for the unmanufacturable shape under the condition of ensuring the complete notification accuracy ratio, and has a great reproducibility value.

## 1. Introduction

Currently, in product design, product descriptions and manufacturing instructions are mostly included independently. Designers often only consider product structure and provinces while ignoring the possible problems of subsequent processing. Failure to fully consider them may lead to the inability to improve capabilities under the existing manufacturing resource environment. In a way to clarify this proposition, it is necessary to perform a manufacturability analysis of the parts in the project layer. Manufacturability analysis refers to thinking about alternatives in the manufacturing process within the product intent, allowing designers to plan the shape and structure of capabilities within the constraints of the manufacturing process and the manufacturing facilitation environment while supporting repetitive management of fixed process information in the manufacturing process analysis and saver constraints. In appendage, this is a prerequisite for able part advancement. A design average that has been analyzed and perfect for manufacturability can greatly reduce the manufacturing cost of the product and deprive the development time. Currently, manufacturability analysis systems are forcibly maintained within the limit of teaching disfavor and basin baseness [1–6]. Factories are bound to adapt when joining new scales or reworking existing behavior, and the arcane science-nourish means only retrains existing plot with new data, can accuse complex manufacturability instructions in new data and has stronger limberness. The plan of a manufacturability analysis is to find and reform indications of nonconformity, and to give a pure purpose of unmanufacturability back to the plotter for modification. Therefore, with the nurture of the mysterious learning system, this wallpaper pressingly teaches the manufacturability of concavity characteristic from the existent data, judges the manufacturability of the hole characteristic, and gives a manifest sense why the arrangement is not manufacturable, so that designers can reduce the fashion.

In view of this, scholars have expounded on the problem of product manufacturability analysis from the aspects of manufacturability analysis mode, system display, and erudition cost. For example, Hu Yanjuan proposed a characteristic-based evaluation method for the manufacturability of self-propelled gears, and introduced the nonbody characteristic modeling and optimization technology based on intelligent algorithms into the manufacturability evaluation system. Yao Chen [7] built knowledge resources for typical aerospace thin-walled material product intentions and products and discussed collaborative operation strategies with the DFM podium. Zhang Jun and Tai Yanfang [8] adopted the manufacturing feature recognition technology and proposed the geometric topology model to establish the manufacturing feature model. Most of the previous studies have adopted the method of paying attention to invaluable and hypothetically abridged rule bases to perform fitting inference, which has a wide range of applications. However, manufacturability analysis systems underpinned by control dishonesty suffer from insufficient flexibility, so some scholars test dense learning algorithms accustomed to manufacturability analysis to weed out data-driven manufacturability judgments.

Three-dimensional dummies are relatively complex, and savvy literature on 3D sight cannot currently be done overnight. Therefore, scholars propose to use voxel, point blackening, and other methods to represent 3D patterns, and customize the sagacious letters method to learn its data. For specimens, Zhang et al.'s [9] Habit 3D-convolutional nerval cobweb (3D-CNN) supports voxel data to identify manufacturing features of parts. Since voxel data are limited by resolution, they cannot specifically represent 3D appearance, and the amount of data is too large. Due to the disorganized nature of point damage data, it cannot be used in time for an exhaustive literature. For this situation, Charles et al. [10] proposed a PointNet grid that can be taught on-the-fly from item blackened data to solve tasks such as object classification and scene segmentation. Wang et al. [11] intend to combine the octree form with full erudition, having an octree-based convolutional neural network (octree-supported CNN, O-CNN) that can be used for feature notification, which can reduce the amount of network training data. In manufacturability analysis of second-hand complete letters, Balu et al. [12] proposed to use a 3D-CNN based on voxel data to dissect the manufacturability of capabilities. The method uses voxels to represent the 3D model, adds the divergence field information of the rectangle to the voxel data, and thus considers the distance between the voxel and the proximal surface of the part, and finally uses these data to induce it. In the same while, Ghadai et al. [13] rise the peripheric exact message of voxels in the voxel data and employed its data to drag the 3D-CNN. These two methods can recite whether the part is manufacturable, but not the reason why the part cannot be manufactured. To sum up, this fallacious reticulation, nurture by the PointNet network construction, erect a pervading and lettered reticulation for the manufacturability analysis of concave features, making full utility of the benefit of thorough academician algorithms, automatically meditation the behavior of shape manufacturability, and distinctive unmanufacturable capabilities. And moment out the arguments for its manufacturability.

## 2. Related Work

There are many factors that affect the machinability of holes. This paper only examines the machining laws of the concave structure and machinability. Reference [13] is concise: for blind holes, the face-to-face ratio of the hollow should be less than 5.0; for through holes, it should be less than 10.0; for holes combined with whiskers, the deviation from the hollow to the feather edge should be larger than the circle of the hole; and for holes involving, the hole bottom should be larger than the hollow radius. According to the above control, parametric modeling technology is used to generate a series of 3D standard-constrained manufacturability caves whose morphological types are not fixed, thus forming an embarrassing graph of manufacturability analysis data.

Since it is difficult to obtain big data of 3D CAD floor plans, this wallpaper adopts a parametric formal modeling system, combined with crack manufacturability management, to generate a manufacturability analysis data set for training the network. The ram judgment is customary CATIA to randomly jointly mine the shape to one-third of the stable size while making sure it has only one hole. Specifically, first, get used to CATIA to create part patterns with cave features and export a design brief with key parameters. Then, supported by the manufacturability principle of the hole, the key parameters of the shape are randomly propagated and written into the design table. Based on the data in the index, secondary development using CATIA tells the interface to grow several response parts dummy. To categorize voids more clearly, each void in the product data is limited to a maximum of one nonmanufacturable component. Then, corresponding to the above rules, it is necessary for CATIA subordinates to develop relevant interfaces to trigger the 3D CAD trend and generate corresponding tickets. It shows the clearance features for different manufacturability categories and the corresponding one-hot codes for that category. This newspaper disseminated a total of 5,000 3D CAD models through the above methods, randomly selected 4,000 designs as training specifications for mystery learning, and finally put 1,000 models into an application as validation.

A given tarnish is a given set of 3D tracks. This time, the nonsolid 3D CAD graphics are all generated by CATIA, and the virtual model is discretized through the significant interface in the CATIA secondary development tool CAA, and the same number of points is maintained in each part through the pattern. Two thousand forty-eight points are extracted per 3D CAD plan and each item contains only coordinate complaints. The affected feature data need to be re-normalized, that is, the coordinate values of all stages are compressed to be between 0 and 1. Due to the perturbation removal and rotation invariance of thorn cloud data, deep learning is not immediately accustomed. The carpel of the PointNet network proposed in Science [10] is to explain these two problems. First, the disorder problem is solved by referencing the planetary properties of the point blackening data through the worn max pooling technology. The max pooling descending window looks from the input feature plane sphere and generates the highest view of each grid and its role.

Downsampling the shape graph to reduce the size and thus the number of parameters; 2. Perform form lineage. Second, the PointNet network guarantees removal and rotation invariance by locating point contamination data. Alignment exercises are done by teaching a data transformer mesh (T-Net) to own the transformation spreadsheet and double the input data to achieve the transformation of the input data. Therefore, this paper takes the PointNet grid as the basic structure and transforms it to study the manufacturability considerations. The point cloud annoyance of hole feature manufacturability analysis is mainly stable T-Net and feature extraction network. The service of the two data transformation networks is to transform the input data and intermediate feature data to a height that is particularly suitable for network learning, while the responsibility of the formal descent network is to perform layer-by-layer shape extraction data on the specified cloud. It has several 2D convolutional bases and a large number of normalization layers worn in the ReLU excitation office (1). Then, add a SpatialDropout2D band [14] and complete the max pooling transformation. The end product level consists of 4 fully integrated courses, 3 Dropout belts, and a Flatten sofa. Compared with PointNet, this paper adds Spatial Dropout2D lift after the 2D convolution sill in the formal extraction plexus to reduce overfitting. Usually, in the preconvolutional band of deep letter grids, whose boundary pixels in the feature mappemonde are strongly correlated, and symmetric dropout techniques will fail to activate regularization. In contrast, the SpatialDropout2D bed in this wallpaper randomly drops the entire 2D feature map, equivalent to dropping several elements. Therefore, Spatial Dropout2D couch will compensate for the independence between shape depictions and be more in line with the mesh in this paper. At the same time, to improve the recognition accuracy and also to deepen the depth of character, a threshold of complete connectivity is added when the network dies, and the normalized exponential function is used as the utility of the activation service. Equation (2) is a normalized exponential activity (Softmax) that reduces any *K*-dimensional royal vector *z* to another *K*-dimensional real vector *σ*(*z*) such that each chemical element in *σ*(*z*) is between 0 and 1. Ramble, the calculation of all elements is 1, where *zj* and *σ*(*z*)*j* represent the *j*th water of vector *z* and vector *σ*(*z*), respectively, relative. The data cooled by multiple sensors can be stored using big data warehousing technology, and the data can be mined through the wear-and-tear neural network algorithm program and crowd algorithm rules. Understanding the decision-making system can determine the operating attitude of the processing system if a storage failure state in the manufacturing process is determined. Adjustment; if it is necessary to adjust the entire process flow and product flow, the production direction can be temporarily closed, and the production will continue after the product and program are optimized to ensure the processing quality of the product.

## 3. Our Method

In the process of geo-mechanical capabilities, in a system with a clear understanding of processing and manufacturing, the analog-digital mint can be combined with the physical factory. Modeling, process instructions, and bump instructions are extended from second-hand analog and digital manufacturing plants, and product advancement and manufacturing are carried out by the second-hand existing intelligent equipment and machine-controlled production lines. During the progress and manufacturing process, the information about the processing and manufacturing delay can also be fed back to the intelligent control terminal, and the process and protrusion instructions can be corrected by using the analog and digital bloomery to improve the processing quality. In a skilled manufacturing process of the mechanical capabilities of the globe, in a system with an increased degree of automation, the working process can be monitored by remote true repeat monitoring. When an unthought-out bankruptcy or procedural industry problem is discovered for a machine, propositional revelation is immediately fed back to understanding care and control systems to adjust protrusions or treatment plans to correct protrusion effects. In the aqiqiy-delay supervision process, the process of an artificial neural network can be used, and the parsing algorithm of the unreserved influence database can be used to distinguish the tokens that the bicycle may already exist or grow sorted. The basic principle is: suppose the intelligent neural network measures the weakness vector *G* = [*G*1i, *G*2i, ⋯, *Gm*i], the desired confidence weight vector is *z* = [*z*1i, *z*2i, ⋯, *zm*i], the corresponding combination of subnets is N*n* = [NN1, NN2, ⋯, NN*n*], thus forming the fault matrix G and the confidence weight matrix *z*, append the dependency spreadsheet to each secondary spider web.

Or for any fusion rise gi greater than a certain threshold, a failure may occur. With this in mind, real-time oversight of the parts custodian's prosecution for fault is possible. When a breakdown occurs, the attitude of the times to automatically sue needs to be adjusted to correct for the particularity of handling. During processing, cognitive decision-making of the auditory ossicles is achieved using the cognitive diagnostic process of bicycle failure or processing quality. In the exchange processing of rural mechanical capabilities, the state parameters of the workpiece and the epigenetic type of the workpiece are collected and taught through sensors, and the tip is transmitted to the central processor for data analysis. The neural network defect diagnosis algorithm program is customized and determined. There are no weaknesses. If there is a fault, the rules are sent directly to the inspection system; if there is no shortage, regulation can continue. With the continuous development of electronic computer hardware and software systems, the emergence of tainted platform technologies, virtual compositions, moral narratives, and potentially camouflaged mechanical products become options. Using a cloud platform and enabling fake software, it is even possible to fake a running farm machine, as well as the training of a Georgia machine. Through the feedback of false data, more technical data allusions can be provided for the design of agricultural machinery, and the optimization of products can be realized before the production of fruit functions. In the intelligent manufacturing process of agricultural machinery parts, the corrosion platform can play an important role in simulation. Because in the process of 3D modeling development, enabling assembly and similarity calculation product capabilities require the comprehensive loading capacity and running speed of electronic computers, and the blackening platform adopts enabling shared storage and collaborative similarity calculation, which is very important. Largely dismissed. Computer behavior. Loading capacity and computing speed provide viable computer resources for understanding the manufacturing of rural mechanical components. Using the quick measure of the blackening scheme data processor, a practical fork of the 3D special-shaped tool can be established, and the confrontation between the tool and the workpiece can be concealed during the 3D machining of the George mechanic ability, and the machining process can be optimized. After completion, record the physical school shift for the procedure. The practicalness of potential steal behavior software UG can go beyond the moral machining of rural mechanical parts. In counterfeit software, it is the only requirement to devise a blank model with formability, then select the appropriate library to utility agreeing to the eminent processing parameters, and then accomplish the potential alikeness of the processing procedure and assimilate to the processing program. Border. Through practical feint, the correct doll passing for anapophysis can be mastered, the processing results can be optimized through backer-deed march data, and workpiece instances can also be gained.

In general digital copy processing, you must preprocess your own data, including monochrome, smoothing, sharpening, and thresholding. In this paper, the detection of local sharpness is very important for the later GA-CNN algorithm rule failure classification, and edge discovery processing is required. The study is contained within a 3 × 5 area, assuming that the sharpening of the curve is delineated by *y* = *a* + *bx* + *cx*^2^. A convolutional neural network (CNN) is a forward grid (9) whose fret structure is mainly decomposed into input, hidden, and output layers. Hidden layers include convolutional layers and full layers. The input layer is used for en features and can handle multidimensional data. The convolutional layer performs feature extraction on the input data and suppresses the manifold convolution kernel. The parameters of the volume layer include the dimensions of warp kernel, intersection, and padding, which together define the specifications of the product, forming a description of the convolution process. The entire floor is dominated by taste. The output layer produces per-pixel classification springs instantaneously.

## 4. Experimental Validation

Based on the cognitive manufacturing system, the combined production line of George Machinery products can produce machine-like performance, and in the unmanned workshop, George Machinery can manufacture the automatic assembly of the ability. In the perceptual production process of agricultural machinery, construction data can be applied to various aspects of the production result. The mining and processing of massive data is also a very important link. Reasonable processing of construction data can save more intense and important costs for the processing and manufacturing process of products and improve fruit efficiency.

In addition to the robotic-like assembly capabilities of agricultural machinery, the combination of flax parts can also be used in more intelligent manufacturing systems. When processing tractor panels, some capabilities that cannot be shredded need to be accomplished through application technology. Manual waving is not only inefficient but also inefficient. And the precision is not as good as the robot automatic welding technology, the application of the intelligent manufacturing system makes the robot's ability to manipulate the tractor very simple. The intelligent automatic rifle processing technology can greatly improve the processing efficiency and ensure the processing quality and high-quality products before the ability description. Optimization also entails optimizing the procedural handling of the product and the resulting performance after narrative, moderately preparing for the uplift technology and process flow. If a compact shape tool is used for processing, the result in the optimization process will inevitably require repeated processing and labor, with a high-speed charging and durable motorcycle; if the simulation experience is used to simulate the processing process and inspect the product, it can effectively improve efficiency and cost reduction. The virtual manufacturing system can use the virtual clothes bowl to imitate the processing process of the parts, and can also observe the movement of the machine during the processing process, can avoid interference between the workpiece and the clothes, etc., and can provide a safe data reference. For solid bicycle tool processing.

3D modeling software UG is a way to design agricultural machinery capabilities. The deduction usage and interface provided by UG is the habit of writing callback functions, and the parameterization scheme of agricultural machinery parts is supported by templates. The parametric design of precision mechanical parts is actually to modify the size parameters of the parts in the learned foundation and examples to coordinate with the design requirements so that the arrangement of the templates and the size can perceive the specified requirements of modern capabilities. Part parametric design process. When optimizing the capability parameters supported by data mining during pregnancy, the capability optimization subsystem is a way of proving the point, line, boundary, and other instructions of the capability model, and then the massive data mining subsystem is interested in training the parameters' ability. The software of the whole system is compiled into ∗.dll and ∗.dlg files, and the concrete realization saver is shown in the following. Taking the rural roadheader's capability sketch as an example, the reliability of the agricultural machinery digital planning system has been verified. Click “Bushing” in “Case Inference Model” on the tenzel donzel of the system, the system will automatically jump to the action inference design interface; then, the designer can start the “Bushing” specification according to the design requirements to get the “Bushing” ‘s display. Drawing. After the action inference model is sculpted, the integral parameters may not be of final quality. At this point, you can capture the “big data mining model” to polish the component parameters, and the system will automatically save the model and display the 3D fashion on the interface.

To support the effectiveness of the reinforcement learning-based manufacturability analysis process for fracture shapes in this paper, quantitative and qualitative comparisons with learning methods [12–17] and belles-lettres [13] are as follows. Both references [12] and [13] voxelize a 3D CAD mold and use the extracted voxelized data to induce a 3D-CNN built from it. The amount of data is much larger than that required for training point sully plexus in this paper. (2) The methods in references [12] and [13] can only try whether the hole shape can be made, but it cannot be avoided manually. The two methods in this paper overcome this problem. (3) The confirmation accuracy rates of the methods in references [12] and [13] are 83.1% and 73.5%, respectively, which are lower than the two methods defined in this paper.

Compared with the usefulness of the fictional 3D-CNN in this article, the details netting supported on the detail cloud data has industry advantages: (1) the amount of point cloud data is much smaller than the amount of voxel data, which is 2.1% of the amount of voxel data; (2) 3D convolution is expensive. In this paper, we induce voxel data of 100 clocks, choose about 3000 s, and perform 210 training sessions on the point-colored data, which only takes 4500 s. The point cloud data genre can hold a lot of ages; (3) voxelize parts, which would leave the integrated count of the grid in a fruitless state (the interior of the section is indeed empty) and not suitable for convolving it into intrinsically useful information. The feature cloud data are all extracted from the epigenes of the parts, so this problem does not hold; (4) since the shape of the hollow feature utility in this paper is relatively simple, the 3D-CNN based on voxel data has a correction in the manufacturability analysis logo, verifying authenticity can deceive 94.5%. When the imagination of the part is complex, the voxel data will not be able to show some specific shapes. It works better only by voxelizing the parts with high disentanglement, but at this time, the volume of the voxel data grows cubically. The amount of point damage data is linearly related to the entanglement of the part. If there is a lack of progress in complex capabilities, the specified amount of cloud training data is much smaller than the amount of voxel data.

## 5. Conclusions

In the design of the manufacturing system of agricultural machinery components, cloud platform technology and virtual simulation software are introduced to realize the intelligent decision-making of the manufacturing system. The virtual resource sharing and collaborative parallel computing of cloud platform technology are used to provide virtual processing and virtual assembly of complex parts. The computing resources are provided, and the machining of parts and the virtual assembly test are realized by using the simulation virtual software. Taking the virtual manufacturing of complex parts of agricultural chassis as an example, the cloud platform and virtual simulation software were used to successfully realize the virtual processing and virtual assembly of products, which provided an important reference for the research on new processing methods of agricultural machinery parts.

## Data Availability

The data can be obtained by requesting the correspondence author.
